# Aurora kinase-C-T191D is constitutively active mutant

**DOI:** 10.1186/1471-2121-13-8

**Published:** 2012-03-26

**Authors:** Jabbar Khan, Sanaullah Khan, Sobia Attaullah, Ijaz Ali, Shahid Niaz Khan

**Affiliations:** 1 Department of Biological Sciences, Gomal University Dera Ismail Khan, Dera Ismail Khan, Pakistan; 2 Institute of Genetics and Development, University of Rennes1, Rennes1, France; 3 Department of Zoology, Kohat University of Science and Technology, Kohat, Pakistan; 4 Department of Zoology, Islamia College Peshawar (A Public Sector University), University Campus, Jamrod Road, Peshawar 25120 Khyber Pakhtunkhwa, Pakistan; 5 Institute of Biotechnology and Genetic Engineering, Khyber Pakhtunkhwa University of agriculture Peshawar, Khyber Pakhtunkhwa, Pakistan

**Keywords:** Aurora-C, Oncogene, Centrosome, Multinucleation, Tumour

## Abstract

**Background:**

Aurora kinases (Aurora-A, B and C) belong to a family of conserved serine/threonine kinases which are key regulators of cell cycle progression. Aurora-A and Aurora-B are expressed in somatic cells and involved in cell cycle regulation while aurora-C is meiotic chromosome passenger protein. As Aurora kinase C is rarely expressed in normal somatic cells and has been found over expressed in many cancer lines. It is suggested that Aurora-C-T191D is not hyperactive mutant.

**Result:**

Aurora-C-T191D variant form was investigated and compared with wild type. The overexpression of Aurora-C-T191D was observed that it behaves like Aurora-C wild type (aurC-WT). Both Aurora-C-T191D and aurC-WT induce abnormal cell division resulting in centrosome amplification and multinucleation in transiently transfected cells as well as in stable cell lines. Similarly, Aurora-C-T191D and aurC-WT formed foci of colonies when grown on soft agar, indicating that a gain of Aurora-C activity is sufficient to transform cells. Furthermore, we reported that NIH-3 T3 stable cell lines overexpressing Aurora-C-T191D and its wild type partner induced tumour formation when injected into nude mice, demonstrating the oncogenic activity of enzymatically active Aurora kinase C. Interestingly enough tumour aggressiveness was positively correlated with the rate of kinase activity, making Aurora-C a potential anti-cancer therapeutic target.

**Conclusion:**

These findings proved that Aurora C-T191D is not hyperactive but is constitutively active mutant.

## Background

Aurora kinases are a conserved family of serine/threonine kinases that are pivotal to the successful execution of cell division. Three Aurora kinases (Aurora-A, -B, and -C), which share sequence homology in their central catalytic kinase domains, have been identified in mammals [1]. All the three mammalian Aurora kinases are implicated as mitotic regulators and due to their elevated expression profiles detected in many human cancers, have generated significant interest in the cancer research field.

Aurora-C is predominantly expressed in the testis [2,3] and is mainly restricted to meiotically dividing spermatocytes [4] and mouse oocytes [5]. Aurora-C is also associated with inner centromere protein (INCENP) in male spermatocytes. Moreover, it is reported that overexpressed Aurora-C kinase behaves like a dominant negative kinase for Aurora-B leading to a cytokinesis defect [6]. Aurora-C disrupts the chromosome passenger protein complexes necessary for cytokinesis. Aurora-C can fulfil the role of Aurora-B in centromere assembly, kinetochore- microtubule attachment, the spindle assembly checkpoint and cytokinesis and, thus, possibly, Aurora-C regulates mitosis by the same mechanisms as Aurora-B in those somatic tissues in which it is overexpressed. Additional potential roles for Aurora-C in somatic tissues could include cooperative or modulating functions in mitosis, or non-mitotic functions such as gene regulation via phosphorylation of histone H3 [7]. Overexpression of Aurora-C in cancerous tissues and cell lines also raises questions about its potential role in carcinogenesis and its effect on the proliferative capacity of tumour cells [8,9]. The expression levels of Aurora-C, Aurora-B and Aurora-B splice variants are commonly altered in tumour cell lines and tissues [10-13]. These alterations in expression have been associated with tumourigenesis, tumour metastasis and tumour aggression. Aurora kinase inhibition by small molecules has been intensively studied recently as a possible cancer therapy [10,14-18].

It is reported that Aurora-C-T191D is hyperactive mutant and its relative activity is sevenfold higher than the activity of Aurora-C-WT [19]. But we report that Aurora-C-T191D is not hyperactive but is constitutively active and behaves exactly like its partner Aurora C-WT.

## Methods

### Construction of vectors

Human aurora-C cDNA was obtained from pET21b-aurora-C [6] by *BglII/EcoRI *digestion and inserted into pEGFP-C3 plasmid (Clonetech USA). Green fluorescence protein (GFP) -aurC-WT DNA was used as a template to obtain K72R, expressing kinase dead GFP-tagged aurC and GFP-aurC-T191D, expressing the constitutively active GFP-tagged aurC by double PCR site directed mutagenesis (Quick change site-directed mutagenesis kit, Stratagene USA), following manufacturer's instructions. The GFP-alone empty vector pEGFP-C3 was used as a control.

### Cell line and transfection

Mouse NIH-3 T3 cells were used in all experiments. Cells were grown in Dulbecco's Modified-Eagle Medium (DMEM) (Gibco USA) containing 10% Fetal Bovine Serum- (PAA France) and 1% Penstrep (GIBCO- 10000 units/ml penicillin + 10000 units/ml streptomycin). Cells were transfected in Lipofectamine™ 2000 transfection reagents (Invitrogen USA) with GFP-aurC-WT, GFP-aurC-CA, GFP-aurC-KD and GFP-alone plasmid DNA, following manufacturer's instructions. For establishment of stable cell line, 800 μg/ml Geneticin G-418 (PAA France) was added in culture media, changing the media twice a week. Clonal selection was performed after 14 days, keeping the cells under continuous pressure of Geneticin G-418.

### Kinase assay

Equal number of stable Cells of GFP-aurC-WT, GFP-aurC-CA, GFP-aurC-KD and GFP-alone were lysed in L-buffer (1% NP40, 250 mM NaCl, 5 mM EDTA, 50 mM NaF, 20 mM Tris-HCl pH 7.5, 1 mM AEBSF, 0.2% Okadaic Acid, Protease inhibitor cocktail (Roche Germany) and 1 mM Na_3_VO_4_). Cell lysates were sonicated and incubated on ice for twenty minutes. The lysates were centrifuged at 13000 rpm for 15 minutes and supernatants were pre-cleared with protein G-sepharose beads (GE Healthcare USA) for twenty minutes at 4°C. The pre-cleared lysates were incubated with 5 μg of Anti-GFP antibody (Roche) and protein G-sepharose beads for two hours at 4°C. The lysates were again centrifuged at 13000 rpm for five minutes at 4°C and the pellets were washed three times with L-buffer containing 500 mM NaCl. The pellets were resuspended in L-buffer and divided into three aliquots, one for kinase assay, on aliquot for western blotting and the third aliquot was saved as a backup at -20°C. The aliquots to be used for kinase assay were washed three times with kinase buffer (50 mM Tris-HCl, pH 7.5, 25 mM NaCl, 10 mM MgCl_2_, 0.1% Triton).

The pellets were resuspended in 20 μl of kinase buffer containing additional 1 mM DTT, 10 μM ATP, 5 μCi γ32P ATP 3000 Ci/mmol (Amersham Pharmacia Biotech USA) and 4 μg of histone H3 (Millipore 14-494 USA). The reaction mix was incubated at 30°C for 30 minutes. Proteins were then separated on 12.5% SDS-polyacrylamide gel electrophoresis. The gel was stained with coomassie blue, dried and analysed by a phosphorimager (Molecular Dynamics USA).

### Soft agar assay

Nine clones each of GFP-aurC-WT and GFP-aurC-CA, and four clones each of GFP-aurC-KD and GFP-alone were tested with this *in vitro *transformation assay. 10,000 cells/well in a 6-well plate in triplicate were grown in 2 ml top agar containing 2X DMEM media, 20% fetal bovine serum and 1% agarose. Geneticin-G-418 was added 24 hours after seeding. Media were changed twice a week. Thirty days after seeding, well plates were stained with 0.005% crystal violet dye and the numbers of colonies were counted.

### Immunofluorescence

10^5 ^cells were grown on 12 mm glass cover slips in a 12-well plate. Cells were washed with PBS and fixed with cold methanol for 10 minutes at -20°C. Fixed cells were washed three times with TBS and then saturated with 1%BSA + 0.1%Tween20 prepared in PBS for 1 hour at room temperature. Primary antibodies in 1%BSA + 0.1%Tween20 in PBS were added on the cells (mouse anti-gamma tubulin, GTU-88-T6557, 1:2500 (Sigma USA); rabbit anti-phospho histone H3 ser-10- 06570, 1:1000 (Millipore USA), rabbit anti-GFP- 632375, 1: 2000 (Clonetech USA) for 2 hours at 4°C, on slow agitation and then washed three times for 10 minutes with TBS. The cells were then incubated with secondary antibodies (anti-mouse Alexa-555, 1: 1000; anti-rabbit Alexa-555, 1:1000; anti-rabbit Alexa-488, 1:1000 (Invitrogen USA) for 1 hour at room temperature on slow agitation, protected from light, washed again with TBS, three times for 10 minutes and then mounted with mounting media- Prolong-Gold (Invitrogen USA), containing DNA staining dye, DAPI. Images were collected using Leica DMRXA2 fluorescent microscope with 63× oil immersion Plan-Apochromat numerical aperture 1.32 objective. Photographs were taken using a black and white cool snap ES camera (Roper Scientific Canada) and images were processed using Metamorph Software (Universal Imaging USA). A minimum of 600 cells was counted for each condition.

### Western blotting

Cells were lysed in RIPA buffer (1% NP40, 50 mMTris HCl, pH 7.5, 150 mM NaCl, 0.25% Sodium deoxycholate, 2 mM EGTA, Protease Inhibitor cocktail (Roche USA). Cell lysates were sonicated and cleared by centrifugation at 13000 rpm for 20 minutes. Proteins were quantified by Bradford method (BioRad USA). Cell lysates were boiled for 5 minutes at 95°C in Laemmli sample buffer. Equal amounts of protein samples were loaded onto 10% SDS-PAGE gel for electrophoresis and then transferred onto nitrocellulose membrane. Membranes were blocked with 5% milk-TBST for 1 hour at room temperature and incubated overnight at 4°C with primary antibodies {Mouse anti-GFP, 1:1000, (Sigma USA); Rabbit polyclonal anti-aurC, 1:250, (Zymed USA)}. Membranes were washed three times for 10 minutes each with TBST and then incubated for 1 hour at room temperature with secondary antibodies {(Anti-mouse coupled with HRP, 1:5000; Anti-rabbit coupled with HRP, 1:30000, (Jackson USA)}. Membranes were washed again with TBST as stated above and then revelation was done with chemiluminiscent, Pico or Dura (Pierce USA).

### Tumour growth

Female nude mice of 3 weeks age, housed in microisolator units under controlled humidity and temperature were fed with sterile diet and water. Stable cell clones to be injected were stained overnight with DilC18(3) (FluoProbes USA) prior to injection. Seven million cells of each were injected subcutaneously in the abdominal region of each mouse. Each mouse was injected with two different clones, one on each side of the abdomen. Tumour sizes were monitored every 10 days by direct observation and the day of sacrifice, using Kodak image station 2000 (Kodak USA) by an excitation of 535 nm that detected cells stained with DilC18(3). Images were then analysed, using Kodak Molecular Imaging Software. Tumour volumes were then determined according to the formula, L × W × H × π/6, shown in mm. Mice were sacrificed when the tumour size reached 1-2 mm^3 ^or two months after injection. Tumours were removed, put immediately in liquid nitrogen and then stored at -80°C for further analysis.

### Immunohistochemistry

Ten-micrometer thick frozen sections of tumours or remaining injected cells were cut on a cryostat (Leica, Milton Keynes, UK) and mounted onto uncoated glass slides. Classical Feulgen staining or Hemalin counterstaining were performed. Immunohistochemistry was performed with rabbit monoclonal KI-67 (1.200, Epitomics, clone SP6) and anti-phospho histone- H3 ser-10 (Millipore USA) and anti-HRP (Jackson USA) secondary antibodies.

### Statistical analysis

Non-parametric Mann-Whitney test was performed and the results were considered statistically significant for a p-value under 0.05.

## Results

### Establishment of GFP-aurC stable cell lines

NIH-3 T3 cells were transiently transfected with GFP-aurC-WT (Wild type), GFP-aurC-CA (constitutively active) and GFP-alone. The expression of GFP-aurC protein was controlled by western blotting 24 hours after transfection with two different antibodies, anti-GFP and anti-aurC (Figure 1A, B). GFP-aurC was identified in GFP-aurC-WT, GFP-aurC-CA and GFP-aurC-KD at 65 KDa with anti-GFP and anti-aurC antibodies. This band is not present in GFP-alone samples. However, we identified GFP-alone at 29 KDa only with anti-GFP-alone antibody.

**Figure 1:** **Western blots, showing GFP-aurC and GFP-alone proteins after 24 hours of transient transfection with GFP-alone, GFP-aurC-KD GFP-aurC-CA and GFP-aurC-WT plasmid DNA with mouse Anti-GFP antibody (A) and with rabbit Anti-aurC antibody (B)**. Western blots showing the level of expression of GFP-aurC protein in three stable clones of GFP-aurC-KD (KD1 to KD3), four stable clones of GFP-aurC-CA (CA1 to CA4), three stable clones each of GFP-aurC-WT (WT1 to WT3) and GFP-alone (GFP1 to GFP3) illustrating the different level of expression of GFP-aurC and GFP proteins by different clones. The antibody used was mouse anti-GFP (**C& D**) and anti-β tubulin antibody as a loading control (**E & F**); (**G**) Kinase assay GFP-aurC-WT, GFP-aurC-CA and GFP-alone clones, using histone-H3 as a substrate. (**H 1,2,3,4**) The left column shows DAPI stained cells and the right column shows phosphorylated cells with Histone-H3 ser-10. (**H-1**) GFP-aurC-WT and (**H-2**) GFP-aurC-CA (**H-3**) GFP-aurC-KD. **(H-4) **GFP-alone (**I**) Histogram shows the percentage of cells with phosphorylation on histone H3 of GFP-aurC-WT, GFP-aurC-CA, GFP-aurC-KD and GFP-alone.

Stable cell lines were generated for GFP-aurC-WT, GFP-aurC-CA and GFP-alone. The level of expression of GFP-aurC and GFP-alone proteins was checked in all stable cell clones with anti-GFP antibody (Figure 1C-F). The level of expression was varied from clone to clone.

### Overexpressed GFP-aurC-WT and GFP-aurC-CA are active kinases

Kinase activity of GFP-aurC was controlled *in vitro*, GFP-aurC-WT, GFP-aurC-CA, GFP-aurC-KD and GFP-alone proteins were immunoprecipitated with anti-GFP antibody and histone-H3-ser10 was used as a substrate. Both the GFP-aurC-WT and GFP-aurC-CA showed kinase activity but the GFP-alone did not show any kinase activity (Figure 1G). We also checked the kinase activity of GFP-aurC-WT, GFP-aurC-CA and GFP-alone *in vivo *in stable cell lines and the phosphorylation of Histone H3 was assayed. The number of positive cells for Histone H3-serine-10 phosphorylated was found almost two fold higher in GFP-aurC-WT and GFP-aurC-CA compared to GFP-alone (Figure 1H, I). Four clones were assayed for each condition.

### Overexpression of active GFP-aurC results in abnormal centrosome number and polyploidy

We used γ-tubulin staining, a centrosomal marker to assess abnormal centrosome amplification (more than two centrosomes per cell) and DNA staining (DAPI) to assess multinucleation (more than one nucleus per cell). It was found that the percentage of cells with abnormal centrosome amplification in GFP-aurC-WT and GFP-aurC-CA was almost 5 times higher than GFP-alone in transiently transfected NIH-3 T3 cells (Figure 2A, B, E, F). Same ratio between GFP-aurC-WT and GFP-aurC-CA was found and compared to GFP-alone in stable cell lines. For multinucleation, we found that the percentage of multinucleated cells in GFP-aurC-WT and GFP-aurC-CA was 5 times higher than multinucleated cells in GFP-alone in transiently transfected NIH-3 T3 cells. Same difference in GFP-aurC-WT and GFP-aurC-CA was found and compared to GFP-alone stable cell lines, showing a clear difference between the two populations *i.e*. GFP-aurC-WT + GFP-aurC-CA and GFP-aurC-KD + GFP-alone (Figure 2C, D, E, G). It was showed that overexpression of active GFP-aurC results in both abnormal centrosome amplification and multinucleation.

**Figure 2:** **Abnormal centrosome amplification and multinucleation**. The immunoflorescent microscopy images **(A-G) **show abnormal centrosome amplification and multinucleation observed in GFP-aurC-WT, GFP-aurC-CA with negative control GFP-alone. **(A&B) **more than two centrosomes/cell appeared as white dots with anti-γ tubulin staining in GFP-aurC-CA and GFP-aurC-WT respectively. (**C**) and (**D**) show multinucleation (more than one nucleus/cell in GFP-aurC-CA and GFP-aurC-WT respectively. **(E) **Two centrosomes per cell and only one nucleus/cell in G_2 _phase of GFP-aur-KD. **(F) **histogram showing the percentage of cells with more than 2 centrosomes/cell of 96 hours after transient transfection in GFP-aurC-CA, GFP-aurC-WT and GFP-alone cells. **(G) **histogram shows the percentages of multinucleated cells of 96 hours after transient transfection in GFP-aurC-CA, GFP-aurC-WT and GFP-alone.

### Aurora kinase C and in vitro transformation

The ability of GFP-aurC was assessed to transform cells in soft agar assay with GFP-aurC-WT and GFP-aurC-CA, and GFP-alone NIH-3 T3 stable cell clones. Nine clones each of GFP-aurC-WT and GFP-aurC-CA and four clones of GFP-alone were tested for growth on soft agar (Figure 3A, B). All the clones of GFP-aurC-WT & GFP-aurC-CA formed a large number of foci of colonies. In contrast, stable cell clones of GFP-alone formed negligible number of small colonies. The data showed that only active overexpressed GFP-aurC has the potential to transform NIH-3 T3 cells.

**Figure 3:** **Soft agar assay, tumour formation and immunohistochemistry**. **(A) **Foci of colonies of GFP-aurA, GFP-aurC-CA, GFP-aurC-WT stable cell lines and very negligible number of very small colonies of GFP-alone in soft agar assay. **(B) **Histogram of the average number of colonies. **(C) **Visualization of the tumours formed by injecting GFP-aurC-CA and GFP-aurC-WT stable cell lines, and the remaining injected cells of GFP-alone on the day of sacrifice using Kodak image station 2000. **(D) **Rabbit monoclonal KI-67, a proliferation marker from late G_1 _to M-phase staining **(E) **anti-phospho histone-H3 ser-10 (Millipore) and anti-HRP (Jackson) secondary antibodies and **(F & G) **Feulgen staining showing prometaphase defects, metaphase defects, lagging chromosomes at anaphase, and cytokinesis defect.

### Aurora kinase C and in vivo transformation

To test whether NIH-3 T3 cells overexpressing GFP-aurC were able to induce neoplastic transformation *in vivo*, eight clones each of GFP-aurC-WT and GFP-aurC-CA and four clones each of GFP-alone were injected (seven million cells of each clone) subcutaneously in Swiss nu/nu mice. Tumours sizes were monitored every 10 days after injection by both direct and indirect measurements. The direct method used was measurements by vernier calliper and the indirectly through fluorometry in live mice. Cells stained with DilC18 (3) dye were excited through skin and the emission signals were used to calculate tumour sizes. We observed a correlation between tumour volumes (Figure 3C-G).

The proliferation status of cells within tumours was analyzed after sacrifice by using different markers. For Ki-67 (a proliferation marker from G_2_/M phase), more than 60% of cells overexpressing GFP-aurC-WT and GFP-aurC-CA were positive for Ki-67 but less than 2% of the injected cells of GFP-alone were positive for Ki-67 (Figure 3D). Feulgen staining of tumours induced by GFP-aurC-WT and GFP-aurC-CA showed abnormal figures of mitosis such as abnormal prometaphase (92%), abnormal metaphase (90%) (Figure 3F) lagging chromosomes (85%) and cytoplasmic bridges (80%) (Figure 3G). No such types of abnormalities were observed in cells overexpressing GFP-alone.

Immunostaining of phosphor-histone H3-serine-10 was used to evaluate the percentage of cells in M-phase. More than 16% of cells overexpressing GFP-aurC-WT or GFP-aurC-CA were histone H3 positive whereas less than 2% of cells overexpressing GFP-alone were positive for histone H3 (Figure 3E). Thus the histological analysis of these tumours confirmed high proliferation rate of both GFP-aurC-WT and GFP-aurC-CA and chromosomal abnormalities.

## Discussion

All the three members of Aurora kinase family have been detected in human cancers when they are overexpressed [10-12]. In this study, whether or not aurora-C-T191D mutant is constitutively active, was in question. We compared the potential to induce cell growth in soft agar and tumour of stable cell lines overexpressing GFP-aurC-WT, GFP-aurC-T191D (GFP-aurC-CA expressing the constitutively active GFP-tagged aurC) and GFP as a control.

We showed *in vitro *kinase assays that the relative activity of histone H3 phosphorylation by GFP-aurC-CA was the same as that by GFP-aurC-WT (Figure 1G-I). These results are in contrast to those previously described [20]. This might be due to the reason that we used mouse NIH3T3 cell line. The GFP-aurC-KD did not phosphorylate Histone H3.

Abnormal expression of Aurora kinases causes abnormal centrosomes amplification and multinucleation [6,17,21]. Both Aurora-A and Aurora-B overexpression phenotypes are aggravated in the absence of active p53 [6,22]. An elimination of the p53-dependent checkpoint may be evoked [23] to explain centrosome amplification and multinucleation induced by Aurora-C. Moreover, overexpressed Aurora-C kinase behaves like a dominant negative kinase for Aurora-B leading to cytokinesis defect that could explain the multinucleation phenotype observed in Aurora-C overexpressing cells [6]. We demonstrated that the overexpression of only active GFP-Aurora-C-CA or Aurora-C-WT induces centrosome amplification and multinucleation (Figure 2).

Although all Aurora kinases are found overexpressed in cancer cells, their direct implication in oncogenesis varies. During interphase Aurora-C localizes to the centrosomes just like Aurora-A, both of them demonstrating oncogenic potentials. Moreover, centrosome amplification, a common feature of Aurora-A and Aurora-C overexpression, is a frequent event in almost all types of solid cancer [24-26]. Interestingly, the kinase activity of Aurora-A is not essential for induction of centrosome amplification, however, the oncogenic transformation requires kinase activity. Aurora-B by itself cannot induce transformation of cells but augments Ras-mediated transformation [27,28]. Aurora-B and -C have overlapping functions and compete each other for their substrates and other chromosome passenger proteins [11]. INCENP and Survivin have stronger affinity for Aurora-B than for Aurora-C [11] but interestingly Aurora-C can complement the functions of Aurora-B in mitotic cells. Although it is likely that the oncogenic activity of Aurora-C is related to its interphase function (Aurora-A like) rather to its mitotic function related to its chromosome passenger behaviour (Aurora-B like) this remains to be deciphered. Similarly we found that the overexpression of Aurora-C induces tumour formation when injected into nude mice, but this needs kinase activity (Figure 3).

It is demonstrated that through both *in vitro *and *in vivo *transformations, overexpression of Aurora-C-CA and Aurora-C-WT in somatic cells has an oncogenic potential and have almost equal relative activity. Thus GFP-aurC-CA is constitutively active kinase mutant, at least in mouse NIH-3 T3 cells, and not hyperactive mutant as has been described earlier in Hela cells and in U2OS cells. Here we used human Aurora-C gene in mouse NIH3T3 cells that needs further to be explored, at least mouse Aurora-C gene in mouse cells.

## Conclusion

On the basis of above stated results and analysis, we thus concluded that at least in NIH-3 T3 cells, the human Aurora C-T191D is constitutively active mutant, and not hyperactive mutant.

## Competing interests

The authors declare that they have no competing interests.

## Authors' contributions

JK designed and performed the experiments, SK participated in discussion of the data and draft of the manuscript. SA, SNK and IA review the manuscript. All authors read and approved the final manuscript.
